# Effect of Mobile Internet Technology in Health Management of Heart Failure Patients Guiding Cardiac Rehabilitation

**DOI:** 10.1155/2022/7118919

**Published:** 2022-02-24

**Authors:** Tao Liu, Mei Liu

**Affiliations:** ^1^Cardiovascular Internal Medicine, Hebei Petrochina Central Hospital, Langfang 065000, China; ^2^Nephrology Department, Hebei Petrochina Central Hospital, Langfang 065000, China

## Abstract

In this paper, we are going to explore the effect of mobile Internet technology in health management for the heart failure patients with cardiac rehabilitation. To implement and evaluate its effects in real environment, a total of 60 heart failure patients were divided, preferably in random fashion, into two groups of 30 cases, i.e., control and observation groups. The former group has received the routine home cardiac rehabilitation after discharge, and the latter group, i.e., observation, has received home cardiac rehabilitation based on mobile medical technical guidance after discharge. The 6 min walking test, Minnesota Cardiac Dysfunction Quality of Life Scale score, cardiac function index, and cardiac rehabilitation training compliance were matched between these groups specifically before and after the intervention. After 12 weeks of intervention, the 6 min walking test, Minnesota Cardiac Dysfunction Quality of Life Scale score, B-type natriuretic peptide of N-terminal, end-diastolic diameter preferably left ventricular, left ventricular ejection fraction, and compliance of training, specifically in the observation group, were better than the control group whereas statistically significant differences were observed, i.e., *P* < 0.01. Home cardiac rehabilitation guided by mobile Internet technology can improve the function of cardiac, exercise tolerance, life's quality, and compliance of patients with heart failure.

## 1. Introduction

Heart failure (HF) is a group of complex clinical syndromes in which ventricular filling or ejection ability is impaired due to any abnormality of cardiac structure or function [1]. Symptoms and signs of heart failure are stable for more than one month, which is called chronic stable heart failure. Heart failure is a severe and terminal stage of various heart diseases, and there are about 230 million patients with heart failure in the world [2]. The prevalence rate of heart failure in China is about 0.9% [3]. Currently, heart failure cannot be cured, and the 5-year survival rate is similar to that of malignant tumors. As an effective way to improve the prognosis of heart failure, exercise rehabilitation was started in the late 1970s [4] which is American college of cardiology foundation and American heart association [5]. Up to now, most Western developed countries have established professional teams for exercise rehabilitation of heart failure, developed relevant operating guidelines or expert consensus, and have relatively perfect community medical environment and hospital home remote monitoring technology. The clinical practice of exercise rehabilitation therapy for heart failure is becoming increasingly popular [6]. However, exercise rehabilitation in patients with heart failure is still in its primary stage in our country, the vast majority of cardiac rehabilitation nursing departments have not been developed, and the competent department of health of both, or cardiovascular physician, nurse, and awareness in rehabilitation treatment for heart failure, combined with community development are not perfect, and most of the patients' contact with the hospital ended after discharge [6, 7]. Although the safety and effectiveness of exercise rehabilitation in patients with heart failure have been proved, most patients with heart failure in China have not benefited from exercise rehabilitation. Therefore, it has become an urgent problem to guide cardiac failure patients to exercise rehabilitation after discharge.

Home, as one of the alternative places for exercise rehabilitation for patients with heart failure after discharge, not only saves resources but also is simple and easy to participate in, which is conducive to the long-term persistence of patients [8]. Home exercise rehabilitation may be a choice with low cost and high efficiency [9]. Studies have confirmed that exercise rehabilitation for patients with heart failure at home has the same effect as exercise rehabilitation in the outpatient department, but the compliance of exercise at home is higher than that in the outpatient department [10]. Mobile medical technology is essentially a medical and health management app supported by smartphones and other mobile terminal systems, providing a new way for family cardiac rehabilitation guidance. At present, cardiac rehabilitation for CHF patients in China is still in its infancy and is only carried out in a few areas.

In this paper, we are going to explore the effect of mobile Internet technology in health management for heart failure patients with cardiac rehabilitation. To implement and evaluate its effects in real environment, a total of 60 heart failure patients were divided, preferably in a random fashion, into two groups of 44 cases, i.e., control & observation groups. The former group has received the routine home cardiac rehabilitation after discharge, and the latter group, i.e., observation, has received home cardiac rehabilitation based on mobile medical technical guidance after discharge. The 6 min walking test, Minnesota Cardiac Dysfunction Quality of Life Scale score, cardiac function index, and cardiac rehabilitation training compliance were matched between these groups specifically before and after intervention.

The rest of the article is organized according to the following agenda items where a comprehensive but brief description of every activity is provided.

In Section 2, mobile Internet technology-based mechanism is presented along with a detailed description of the various subparts. In Section 3, various results, which are obtained through extensive experiments, are presented both in textual and graphical format. Finally, concluding remarks are given which is preceded by a detailed discussion section.

## 2. Proposed Mobile Internet Technology-Based Method

### 2.1. Participant

Sixty HF patients admitted to our hospital from June 2020 to May 2021 were selected as the research subjects.

Inclusion criteria are as follows: conforming to the diagnostic criteria of 2014 Guidelines for the Diagnosis and Treatment of Heart failure in China [4], heart function grading II∼III, left ventricular ejection fraction (LVEF)< 45%, stable condition for more than 1 month, equipped with android mobile phone and capable of using a smartphone, and aged 40∼80.

Exclusion criteria are as follows: patients with uncontrolled hypertension, severe ventricular arrhythmia, hypertrophic obstructive cardiomyopathy, aortic stenosis, intracardiac or deep vein thrombosis, severe pulmonary disease, and other reasons for exercise contraindications. This study has been approved by the hospital ethics committee.

### 2.2. Exercise Method

  Control group: After discharge, patients were given routine treatment of HF and family cardiac rehabilitation, including regular administration of G receptor blockers, angiotensin-converting enzyme inhibitors, angiotensin II receptor blockers, aldosterone receptor antagonists, and guidance on reducing body weight, changing dietary habits, and quitting smoking. Before discharge, according to the ECG treadmill test, individualized exercise prescription was formulated according to Bruce scheme or symptom restrictive scheme [5], the form of aerobic exercise of fast walking or jogging was taken, exercise time is 30∼60 min/time, 3∼5 times a week, and the exercise intensity was determined according to the heart rate and Borg self-perceived fatigue rating [6], and the target heart rate during exercise = resting heart rate + (maximum exercise heart rate−resting heart rate) × 0.4, gradually increasing [7]. Family exercise rehabilitation guidance was carried out through telephone consultation or outpatient follow-up.
  Observation group: ofter discharge, on the basis of HF routine treatment, family cardiac exercise rehabilitation training guided by mobile medical technology (sports rehabilitation app) was conducted.

### 2.3. The Software Designed

A smartphone exercise rehabilitation app based on an Android system is designed, which has the following functional modules: data reading module, which can read various exercise data of smart bracelet in real time, such as heart rate, exercise speed, exercise time, and other parameters. Exercise prescription module sets exercise intensity, exercise frequency, exercise time, maximum heart rate, weekly exercise course arrangement, and alarm clock reminder; Exercise guidance module voice prompts current exercise speed, heart rate, acceleration or deceleration reminder, exercise rhythm adjustment, etc. In remote guidance module, the patient's mobile phone app can automatically upload various exercise parameters to the cardiac rehabilitation center of the hospital, and the cardiac rehabilitation center can timely adjust the exercise prescription according to the actual exercise situation of the patient. Health education module regularly receives the rehabilitation education knowledge pushed by the hospital rehabilitation center. The exercise rehabilitation app software is designed by the family cardiac exercise rehabilitation training research team (1 chief cardiovascular physician and 3 nurses with more than 10 years of specialized work experience) and the engineers of the information department, who are responsible for software debugging, operation, and system maintenance.

### 2.4. Family Cardiac Exercise Rehabilitation Training Guided by App

Before the patients were discharged, the nurses in the research team assisted the patients to install the exercise rehabilitation app and taught the patients to use it. In the movement process, the app guides the patients all the way, who were with headphones and a bracelet with functions of monitoring the heart rate with intelligence; according to app voice prompt, there are pace of warm-up exercise, formal sports, and exercise. In the process of formal movement, the software automatically obtain real-time motion in patients with heart rate, and according to the preset target heart rate, combined with patient toil, voice prompts the patient to speed up or slow down. Patients choose exercise time and intensity according to their own situation. The cardiac rehabilitation center provides remote guidance and health education through the online data of various actual exercises fed back by mobile terminals. The rehabilitation team adjusts exercise prescriptions in time by analyzing the feedback data. If the patient does not complete the exercise plan, a remote reminder will be carried out to urge the patient to complete the training.

### 2.5. 6 Min Walking Test (6 MWT)

6 MWT was used to evaluate the therapeutic effect of heart failure. Patients were asked to walk in a straight corridor at the fastest speed they could tolerate, and their walking distance for 6 min was measured. Walking distance <150 m was severe heart failure, 150–450 m was moderate heart failure, and >450 m was mild heart failure [8]. The two groups were tested by two nurses before discharge and at the follow-up of 12 weeks after intervention, and the two walking distances were recorded as the evaluation basis of exercise rehabilitation effect.

### 2.6. MLHFQ Score

LHFQ included 21 questions in physical field (8 questions), emotional field (5 questions), and other fields (8 questions). The Likert 6-point scoring method was adopted. 0 points indicated that heart failure had no impact on patients, and 5 points indicated that heart failure had a serious impact on patients. It indicates that the quality of life of patients with heart failure is worse [9]. Patients in both groups were instructed by nurses to read each question of the scale before discharge and during the 12-week follow-up of intervention. Patients circled the results of each question (0, 1, 2, 3, 4, and 5) and recalled the statistical score of the scale and recorded it.

### 2.7. Cardiac Function Index Examination

Cardiac function indexes of patients in both groups were examined before discharge and at the follow-up of 12 weeks after intervention: N-terminal B-type natriuretic peptide (NT-proBNP), left ventricular end-diastolic diameter (LVEDD), and LVEF were recorded by color ultrasound examination. The effect of exercise rehabilitation was evaluated according to the data mentioned above.

### 2.8. Compliance of Sports Rehabilitation Training

The control group received regular telephone follow-up, and on completion of an outpatient appointment, the patients' exercise prescriptions were asked, and the movement of the group was monitored according to uploaded software to ensure that the background prescribed exercises were completed. The compliance of exercise rehabilitation of patients was evaluated, with more than 80% for good adherence, 50%∼79% for compliance, and below 50% for poor compliance.

### 2.9. Statistical Analysis

We have utilized the SPSS 19.0 software to perform the statistical analysis of data. Measurement data are depicted as (*x* ± *s*) whereas two samples (preferably independent) were utilized to carry out the comparison of intergroup. The *χ*^2^ test was used for counting the data. Grade data were analyzed by *Ridit* with the significance level = 0.05.

## 3. Experimental Results and Evaluation

### 3.1. General Information

The proposed study was approved through the ethics committee of the concerned hospital. Finally, 60 patients were enrolled which have signed the consent and were divided into control and observation groups where each group was assigned 30 patients through a random mechanism (preferably random number table). The control group consists of 18 males and 12 female patients with age (55.27 ± 6.01) years, and 20 patients with grade-II cardiac function and 10 with grade-III cardiac function. The observation group has 17 males and 13 females patients with average age (53.27 ± 7.1) years, and 22 patients with grade-II cardiac function and 8 patients with grade-III cardiac function. We have observed no or zero significant difference in these groups (*P* > 0.05) specifically in the general data.

### 3.2. Comparison of 6 MWT and MLHFQ Scores between the Two Groups

There were no statistically significant differences in 6 MWT and MLHFQ scores between the two groups at discharge (*P* > 0.05). After 12 weeks of intervention, 6 MWT and MLHFQ scores in the observation group were better than those in the control group, with statistically significant differences (*P* < 0.01) (see Table 1).

### 3.3. Comparison of Cardiac Function Index Values between the Two Groups

There was no significant difference in NT-proBNP, LVEDD, and LVEF between these groups at discharge (*P* > 0.05); After 12 weeks of intervention, the index values of NT-proBNP, LVEDD, and LVEF in the observation group were better than those in the control group, and the difference was statistically significant (*P* < 0.01) (see Table 2).

### 3.4. Comparison of Motor Rehabilitation Compliance between the Two Groups

The compliance of exercise rehabilitation in the observation group was significantly higher than that in the control group (*P*=0.001) (see Table 3).

## 4. Discussion

HF patients are prone to shortness of breath, palpitation, fatigue, and other symptoms during activities and often dare not exercise, resulting in decreased exercise endurance. In addition, HF patients have poor self-care ability, recurrent illness, high readmission rate, and great psychological pressure, resulting in decreased quality of life. A meta-analysis of 729 HF patients in 11 randomized clinical studies showed that exercise rehabilitation reduced the risk of death by 39% [10]. With the increasing popularity of mobile terminals such as smart phones, this study designed and taught patients to use sports rehabilitation app to provide online family cardiac rehabilitation exercise guidance and push relevant health self-management knowledge so as to provide online consultation for patients. Wearing the smart bracelet can obtain the heart rate and other sports parameters and can dynamically monitor the patient's heart rate during exercise with good accuracy. In this study, after 12 weeks of home cardiac rehabilitation guided by exercise rehabilitation app, the average distance of 6 MWT in the observation group was significantly better than that in the control group, and the MLHFQ score was significantly lower than that in the control group, with statistically significant differences between the two groups (*P* < 0.01).

NT-proBNP, LVEDD, and LVEF are all used for cardiac function monitoring and prognostic judgment. NT-proBNP as a peptide hormone, by ventricular cardiomyocytes subdivided and reflect ventricular tension and the body ventricular pressure, hormone regulation system, dyspnea degree is directly related, the change of NT-proBNP level can effectively reflect the degree of heart failure. LVEF reflects cardiac contractility and reserve function and increases as cardiac function improves. The results of this study showed that after 12 weeks of family cardiac rehabilitation testing, the observation group NT-proBNP and LVEDD were significantly lower than the control group. LVEF was significantly higher than the control group, and the difference between the two groups was statistically significant (*P* < 0.01), indicating that family cardiac rehabilitation exercise based on mobile medical technology guidance can effectively improve the cardiac function of patients.

Routine home cardiac rehabilitation for HF patients lacks real-time guidance from medical staff and poor compliance, and patients cannot correctly master the amount of exercise, which affects the effect of exercise rehabilitation. The home remote cardiac rehabilitation guided by mobile medical technology can solve most of the obstacles for patients to participate in home cardiac rehabilitation [11]. The background system can read the exercise heart rate, exercise speed, exercise time and other parameters of the smart bracelet in real time and guide the exercise rehabilitation training plan of HF patients in the whole process according to the preset exercise prescription. The amount of exercise in real time was adjusted according to the patient's exercise heart rate to fully achieve the exercise effect. At the same time, the functions of the exercise rehabilitation app, such as automatic reminder, supervision, remote guidance, and the push of cardiac rehabilitation knowledge, make it easy for patients to accept so as to improve the exercise compliance. The results in Table 3 showed that, after intervention, the compliance of exercise rehabilitation in the observation group was better than that in the control group (*P* < 0.01), indicating that home cardiac rehabilitation guided by mobile medical technology can improve the compliance of cardiac rehabilitation exercise in patients.

## 5. Conclusion and Future Directives

As a chronic disease, heart failure has a long time span of health management and a wide range of fields. The traditional medical care model is limited by time and space and cannot provide continuous high-quality health management services for patients. Health analysis is to manage personal health information and evaluate personal health and disease risks. At present, we use mobile Internet technology to carry out personalized nursing and health management for individuals, which has the advantages of convenience, openness, interaction, and real-time. Doctor-patient communication can better supervise and remind patients and provide professional health guidance for patients. The results of the nursing application based on mobile Internet technology in the health management of patients with heart failure show that patients' compliance behavior is better and patients' health literacy is higher. Nursing based on mobile Internet technology has to be implemented to build a new nursing concept, across time and geographical boundaries and to inform the disease knowledge continuously to patients. On the one hand, health education is relatively insufficient to solve the medical information and the increasing contradiction of supply and demand of patients with chronic disease, which leads to heart failure. On the other hand, to ensure that patients undergo health education repeatedly and in stages, the health management effeciency has to be better. In conclusion, the implementation of nursing based on mobile Internet technology can help improve the effectiveness of health management of patients with heart failure and improve the health literacy of patients.

In future, we are eager to extend the proposed mobile Internet technology-based system for the early prediction of heart failure specifically in elder patients with an age factor of 60 plus.

## Figures and Tables

**Table 1:** Comparison of 6 MWT and MLHFQ scores between the two groups.

Group	*n*	6 MWT (m)		MLHFQ score	
		Out of the hospital	12 weeks after intervention	Out of the hospital	12 weeks after intervention
Control group	30	246.57 ± 20.65	289.69 ± 22.62	47.26 ± 6.78	41.27 ± 4.19
Observation group	30	248.58 ± 21.72	347.26 ± 33.27	48.07 ± 5.92	38.65 ± 3.99
*T*		0.698	8.676	0.895	5.671
*P* value		0.445	<0.01	0.373	<0.01

**Table 2:** Comparison of NT-proBNP and cardiac color ultrasound between the two groups.

Group	*n*	NT-proBNP		LVEDD (mm)		LVEF %	
		Out of the hospital	12 weeks after intervention	Out of the hospital	12 weeks after intervention	Out of the hospital	12 weeks after intervention
Control group	30	3057.56 ± 202.36	2287.22 ± 236.86	60.17 ± 7.88	59.26 ± 7.04	35.41 ± 6.17	39.75 ± 5.22
Observation group	30	3088.21 ± 198.52	1566.21 ± 175.98	59.47 ± 6.02	52.88 ± 6.53	36.02 ± 5.12	43.66 ± 4.14
*t*		0.472	16.21	0.366	9.16	0.862	2.896
*P* value		0.689	<0.01	0.877	<0.01	0.426	0.007

**Table 3:** Comparison of exercise rehabilitation compliance between the two groups.

Group	*n*	Good compliance	General compliance	Poor adherence
Control group	30	12	10	8
Observation group	30	5	12	13

## Data Availability

The datasets used and analyzed during the current study are available from the corresponding author upon reasonable request.

## References

[1] Salankar N., Koundal D. (2021). Mian qaisar S. Stress classification by multimodal physiological signals using variational mode decomposition and machine learning. *Journal of healthcare engineering*.

[2] Yong-lin S. U., Jing-kang L. U., Hua G. (2018). *Progress of Tele-Monitoring Exercise Training in Patients with Chronic Heart Failure*.

[3] Kaur M., Kumar V., Yadav V., Singh D., Kumar N., Das N. N. (2021). Metaheuristic-based deep COVID-19 screening model from chest X-ray images. *Journal of Healthcare Engineering*.

[4] Kang Q., Liu W. (2018). Chinese Guidelines for the diagnosis and treatment of heart Failure 2018. *Chinese Journal of Cardiology*.

[5] Ratter J., Radlinger L., Lucas C. (2014). Several submaximal exercise tests are reliable, valid and acceptable in people with chronic pain, fibromyalgia or chronic fatigue: a systematic review. *Journal of Physiotherapy*.

[6] Piepoli M. F., Conraads V., Corrà U. (2014). Exercise training in heart failure: from theory to practice. A consensus document of the heart failure association and the European association for cardiovascular prevention and rehabilitation. *European Journal of Heart Failure*.

[7] Kang T., Wei W. (2014). Consensus of Chinese experts on exercise rehabilitation of chronic stable heart failure. *Chinese Journal of Cardiology*.

[8] He H., Li A., Lin Q. (2015). Chinese expert consensus on exercise therapy for patients with coronary heart disease. *Chinese Journal of Cardiovascular Disease*.

[9] Moughrabi S., Evangelista L. S., Habib S. I. (2013). patients with stable heart failure, soluble TNF-receptor 2 is associated with increased risk for depressive symptoms. *Biological Research For Nursing*.

[10] Keteyian S. J., Piña I. L., Hibner B. A., Fleg J. L. (2010). Clinical role of exercise training in the management of patients with chronic heart failure. *Journal of Cardiopulmonary Rehabilitation and Prevention*.

[11] Ines F., Vanhees L., Dendale P., Goetschalckx K. (2014). A review of telerehabilitation for cardiac patients. *Journal of Telemedicine and Telecare*.

